# On the Effect of Electroacupuncture in Promoting Healing after High Tibial Osteotomy

**DOI:** 10.1155/2022/6428759

**Published:** 2022-03-17

**Authors:** XiangDong Tian, Xia Li, LiQun Zhou, JiPing Zhao, XiaoMin Li, Ye Huang, TianSong Ding

**Affiliations:** ^1^Dongzhimen Hospital, Beijing University of Chinese Medicine, Beijing 100700, China; ^2^Wudang Medical Institute, Beijing University of Chinese Medicine, Beijing 100029, China; ^3^The Third Affiliated Hospital, Beijing University of Chinese Medicine, Beijing 100029, China

## Abstract

**Purpose:**

To explore the clinical effect of electroacupuncture in promoting the healing of the osteotomy area after high tibial osteotomy.

**Methods:**

50 patients with knee osteoarthritis who underwent open wedge high tibial osteotomy (OWHTO) were selected and randomly divided into the observation group and control group. The control group got the common postoperative treatment, and the observation group was added electroacupuncture from the 3rd day after the operation on the basis of the control group. The electroacupuncture acupoints were selected SP10, ST34, ST32, EX-LE2, ST40,KI6, KI3, SP6, and ST41, once a day, and 14 days were a course of treatment. And then we contrasted the index of the Lane-Sandhu X-ray score, the skin incision healing time, the swelling subsided time, Visual Analogue Scale (VAS), Western Ontario and McMaster Universities Osteoarthritis Index Score (WOMAC), and Lysholm in different time.

**Results:**

The Lane-Sandhu X-ray score of the observation group was better than that of the control group at all time points (*P* < 0.05), and the time to achieve bone healing was about 2 weeks earlier than that of the control group. The skin healing and swelling were the subsided time in the osteotomy area. Both were better than the control group, and the difference was statistically significant (*P* < 0.05). The VAS score, WOMAC score, and Lysholm score of the two groups were significantly improved compared with preoperatively, and the difference was statistically significant (*P* < 0.05). The improvement of the observation group's VAS score, WOMAC score, and Lysholm score at 1 week, 4 weeks, and 8 weeks after the end of the treatment course was better than that of the control group, and the difference was statistically significant (*P* < 0.05).

**Conclusion:**

Electroacupuncture can quicken the healing of bone tissue and surrounding soft tissues in the osteotomy area after high tibial osteotomy, and at the same time, it can help the relief of knee joint pain and improve knee joint function.

## 1. Introduction

Knee osteoarthritis (KOA) is a common cartilage degenerative disease which causes a high disability rate [1–4]. It usually occurs in the medial compartment, which often forms medial single-compartment knee osteoarthritis (MSCKOA) and leads to knee varus deformity [5, 6]. High tibial osteotomy (HTO) becomes more and more popular to be a treatment methods of medial compartment knee osteoarthritis, which can effectively relieve knee symptoms and improve knee joint function [7, 8]. Open wedge high tibial osteotomy (OWHTO) is the current mainstream osteotomy method, with a wide range of clinical applications [9].

Although the strong internal fixation of the osteotomy area is the guarantee for the success of the operation, the healed time of the osteotomy is also an important factor to finish the treatment of KOA. Nowadays, allograft bone is used to fill the area to speed up the healing of the fracture area. However, is there an effectively methods such as physical treatment to do it well? We used acupuncture to do it.

In traditional Chinese medicine, acupuncture and moxibustion have been studied [10–12] to promote fracture healing to a certain extent. Electroacupuncture has less relevant reports on the effect of promoting the healing of the osteotomy area after high tibial osteotomy.

In the paper, electroacupuncture was used as an intervention treatment after tibial osteotomy to explore the effect of promoting the healing of the osteotomy area after high tibial osteotomy.

## 2. Methods

### 2.1. Patients

50 patients with MSCKOA were treated in the Department of Minimally Invasive Arthritis of The Third Affiliated Hospital of Beijing University of Chinese Medicine from January 2020 to October 2020. The patients were randomly divided into the observation group and observation group using the randomized envelope method, 25 cases in each group. The difference in baseline data between the two groups was not statistically significant (*P* > 0.05).

The inclusion criteria were as follows: (1) patients with MSCKOA, (2) receiving high tibial osteotomy, (3) age 40 to 70 years old, (4) consciously able to cooperate with treatment, and (5) signed informed consent book.

The exclusion criteria were as follows: (1) knee osteoarthritis and destruction of lateral cartilage; (2) combined with knee gouty arthritis, rheumatoid arthritis, and other diseases; (3) combined with severe diabetes, hypertension and severe liver and kidney insufficiency, and other diseases; and (4) combined with chronic wasting diseases such as tuberculosis and tumors as shown by Table 1.

### 2.2. Treatment Methods

#### 2.2.1. Control Group

Routine rehabilitation program begins after surgery. On the first day after the surgery, the patient underwent an ankle pump exercise. The day after the operation, a knee flexion and extension exercise were performed. The third day after the operation, patient began to walk to the ground with the help of a walker. Two weeks after surgery, the patient walked with the assistance of double crutches. At 8–10 weeks after the surgery, the patient walked autonomously.

#### 2.2.2. Observation Group

On the basis of the treatment of the control group, electroacupuncture treatment was started on the 3rd day after operation. Acupoint selection is as follows: SP10, ST34, ST32, EX-LE2, ST40, KI6, KI3, SP6, and ST41. Acupuncture procedure is to get the patient's cooperation firstly and then mark the right acupuncture points; secondly, next step is to select 0.3 × 40 mm disposable acupuncture needles and then to puncture the needles that is 90° to the skin, and the depth is about 3 cm. After that, the pulse electroacupuncture device (Indy KWD-808-I Changzhou Indy Electronic Medical Equipment Co., Ltd., Su Xie Zhun 20152261330, Figure 1(a)) is connected with the end of the needles separately (Figure 1(b)), selects the stimulus intensity tolerated by the patient, and routinely retains the needle for 30 minutes, once a day. 14 days are a course of treatment.

### 2.3. Observation Indicators

#### 2.3.1. Lane-Sandhu X-Ray Scoring

It is used to evaluate the healing of bone tissue in the osteotomy area.

#### 2.3.2. Incision Healing Time and Lower Limb Swelling Time

The incision healing time and lower limb swelling time were used to evaluate the recovery of soft tissue after osteotomy. The lower limb swelling was evaluated by the difference between the circumference of the thigh and the calf and compared with the healthy limb.

#### 2.3.3. VAS

It is used to evaluate knee joint pain, which is from 0 to 10 points. The larger the score, the more painful it is.

#### 2.3.4. WOMAC

It is used to evaluate knee joint function. The higher the score, the worse the knee joint function.

#### 2.3.5. Lysholm Scale

It is used to evaluate knee joint function. The lower the score, the worse the knee joint function.

### 2.4. Statistical Analysis

Statistical analysis was performed using SPSS22.0, measurement data were expressed as mean ± standard deviation, paired *t*-test was used for comparison within groups, two independent sample *t*-test was used for comparison between groups, and rank sum test was used if the data did not conform to the normal distribution. The count data was tested by the *χ*^2^ test, and *P* < 0.05 was statistically significant.

## 3. Results

Both groups of patients successfully completed the operation without intraoperative complications. Both groups of patients completed the postoperative treatment and were followed up. There was no infection in the two groups after the operation, and no serious adverse reactions occurred after the operation.

The bone healing in the osteotomy area of the observation group was better than that of the control group at all time points (*P* < 0.05), and the time to achieve bone healing was about 2 weeks faster than that of the control group as shown by Table 2 and Figure 2.

The skin healing time of the observation group and the time to reduce swelling were better than those of the control group, and the difference was statistically significant (*P* < 0.05) as shown by Table 3.

At 1 week, 4 weeks, and 8 weeks after the treatment, the VAS score, WOMAC score, and Lysholm score of the observation group and the control group were significantly improved compared with preoperatively, and the difference was statistically significant (*P* < 0.05); the VAS score of the observation group, WOMAC score, and Lysholm score was better than the control group at 1, 4, and 8 weeks after treatment (*P* < 0.05) as shown by Table 4 and Figures 3–5.

## 4. Discussion

### 4.1. Healing Time of Fracture by Some Effective Methods

With the continuous advancement of the concept of enhanced recovery after surgery (ERAS) and the search for comprehensive treatment methods to promote the rapid healing of the osteotomy area, the recovery of knee joint function and relieve pain has attracted more and more attention from clinicians. In order to seek rapid healing of the osteotomy area after THO, we have made efforts to do it.

We used strong internal fixation and bone grafting in the osteotomy area to promote the healing of the osteotomy as other surgeons do. Studies have shown that [13, 14] strong internal fixation materials can promote fracture healing and to make patients to walk as soon as possible, which is conducive to the recovery of lower limb function. Wedge-shaped osteotomy on the medial tibia will lead to a wedge-shaped bone defect area, and the larger the expansion angle, the larger the defect volume, which may increase the risk of nonunion of the osteotomy area. Therefore, it is necessary to perform bone grafting operation [15, 16] to avoid the risk of bone nonunion. However, how to promote the healing of the osteotomy area through other methods is still a big challenge.

### 4.2. Acupuncture in the Healing Time of Fracture

Acupuncture, as a traditional Chinese medicine therapy, has the functions of dredging the meridians, reconciling qi and blood, and promoting blood circulation [17]. Study [18] has found through animal experiments that acupuncture can improve the blood circulation in the fracture area, thereby promoting fracture healing. Du [19] found through clinical research that acupuncture can promote the deposition of minerals and trace elements at the fracture site and accelerate the fracture healing process. Studies have also found that [20, 21] acupuncture can speed up fracture healing by regulating human hormone levels. In addition, acupuncture can also promote fracture healing by regulating the process of bone formation and bone destruction, activating the WNT/*β*-catenin signal pathway protein, and regulating the level of cell growth factors [22].

Electrical stimulation therapy is a type of physical therapy, which has been widely used in clinical practice [23, 24]. Studies have found that [25] electrical stimulation therapy can promote fracture healing by improving circulation and adding bone nutrition. Although the specific mechanism of electrical stimulation to promote fracture healing has not yet been uniformly concluded, relevant basic research and clinical studies have shown that the effect of electrical stimulation on promoting fracture healing is definite [26–28].

Studies have suggested that [29–31] the mechanism of electrical stimulation to promote fracture healing may be that osteoblasts are induced by electrical stimulation to produce a variety of bone growth factors, thereby accelerating fracture healing. Fitzsimmons et al. [32] found in a model study of electrical stimulation of bone tissue that short-term electrical stimulation can promote the secretion of insulin-like growth factor-II (insulin-like growth factor-II, IGF-II) by osteoblasts.

Studies have also found that [33] electrical stimulation can promote the expression of transforming growth factor-*β* (TGF-*β*), BMP2, and BMP4 in osteoblasts, thereby accelerating the process of fracture healing. Kuzyk et al. [34] believed that under the action of electrical stimulation, the originally closed microvessels opened, which enriched the local blood supply, stimulated the proliferation and differentiation of bone cells and chondrocytes, promoted the deposition of mineral calcium, and shortened the calcification time, and reduce osteoclast activity and bone resorption, increase the production of bone tissue matrix protein, and strengthen bone tissue [35].

In addition, the normal effect of the electromagnetic field can also speed up the fracture healing process. The bone structure integrity is heavily influenced by the material properties that are dependent on certain characteristics [36, 37]. Predictive control [38] of diagnosis can contribute to the healing effect.

## 5. Limitation of the Study

This study has its limitations, such as one of the barriers to demonstrating rapid healing of the fracture area in surgical and medical image diagnosis is plate occlusion limiting the evaluation of more points in the fracture area and having an impact on the data.

## 6. Conclusion

We found that electroacupuncture can significantly promote the healing of bone tissue and surrounding soft tissues in the osteotomy area after HTO, which also can speed up the relief of knee joint pain and improve knee joint function. As a clinically effective and simple and inexpensive treatment method, it is worthy to be clinical promotion.

## Figures and Tables

**Figure 1:** (a) Electroacupuncture treatment instrument. (b) Schematic diagram of electroacupuncture treatment.

**Figure 2:** (a) Results of Lane-Sandhu X-ray score in the observation group. (b) Results of Lane-Sandhu X-ray score in the control group.

**Figure 3:** (a) Results of VAS score in the observation group. (b) Results of VAS score in the control group.

**Figure 4:** (a) Results of WOMAC score in the observation group. (b) Results of WOMAC score in the control group.

**Figure 5:** (a) Results of Lysholm score in the observation group. (b) Results of Lysholm score in the control group.

**Table 1:** Comparison of general baseline data between the two groups.

Index	Observation group(*n* = 25)	Control group(*n* = 25)	Statistics	*P* value
Age $\left(\bar{x}\pm s\right)$	64.76 ± 6.07	64.84 ± 8.84	*t* = −0.037	0.970
Gender (male/female)	8/17	6/19	*X* ^2^ = 0.397	0.529
Affected limb (left/right)	11/14	12/13	*X* ^2^ = 0.081	0.777
BMI index $\left(\text{kg}/{\text{m}}^{2},\bar{x}\pm s\right)$	26.37 ± 3.38	28.92 ± 3.59	*t* = −1.475	0.147

**Table 2:** Comparison of Lane-Sandhu X-ray scores of fracture healing between the two groups ($\bar{x}\pm s$, points).

Group	Number	4 weeks	8 weeks	10 weeks	12 weeks	14 weeks	*F*	*P*
Observation	25	2.08 ± 1.08	5.68 ± 1.38	8.72 ± 1.34	12.00 ± 0.00	12.00 ± 0.00	815.810	<0.001
Control	25	1.08 ± 0.70	3.92 ± 1.22	6.96 ± 1.27	9.16 ± 1.21	11.04 ± 6.76	245.814	<0.001
*Z*		-3.417	-3.976	-4.014	-6.310	-5.360		
*P*		0.001	<0.001	<0.001	<0.001	<0.001		

**Table 3:** Comparison of soft tissue healing between the two groups.

Group	Number of cases	Incision healing time	Swelling time
Observation group	25	10.88 ± 1.86	10.24 ± 1.81
Control group	25	13.40 ± 1.87	13.52 ± 2.04
*t* value		-4.782	-6.008
*P* value		<0.001	<0.001

**Table 4:** Comparison of follow-up data between the two groups ($\bar{x}\pm s$, points).

Index	Point in time	Observation group (*n* = 25)	Control group (*n* = 25)	Statistics	*P* value
VAS	Preoperative	7.92 ± 1.04	7.52 ± 0.87	*z* = −1.345	0.179
	1 week after treatment	2.20 ± 0.96	3.08 ± 0.86	*z* = −3.090	0.002
	4 weeks after treatment	0.80 ± 0.71	1.48 ± 0.77	*z* = −2.943	0.003
	8 weeks after treatment	0.44 ± 0.51	1.04 ± 0.79	*z* = −2.771	0.006
	*F* value	371.121	436.465		
	*P* value	<0.001	<0.001		

WOMAC	Preoperative	117.92 ± 18.13	120.40 ± 17.70	*t* = −0.489	0.627
	1 week after treatment	95.15 ± 2.44	99.68 ± 3.66	*t* = −5.135	<0.001
	4 weeks after treatment	80.36 ± 2.29	87.12 ± 2.13	*t* = −10.815	<0.001
	8 weeks after treatment	73.96 ± 4.39	80.36 ± 2.31	*t* = −6.450	<0.001
	*F* value	184.189	144.782		
	*P* value	<0.001	<0.001		

Lysholm	Preoperative	48.68 ± 5.18	48.08 ± 4.00	*t* = 0.459	0.649
	1 week after treatment	78.80 ± 2.02	65.00 ± 4.61	*t* = 13.709	<0.001
	4 weeks after treatment	90.88 ± 1.86	83.80 ± 3.16	*t* = 9.655	<0.001
	8 weeks after treatment	92.20 ± 2.04	87.52 ± 2.79	*t* = 6.776	<0.001
	*F* value	760.937	755.786		
	*P* value	<0.001	<0.001		

## Data Availability

Data are available on request from the authors due to privacy/ethical restrictions.
